RETRACTED

# Nursing Effect of Health Monitoring System on Elderly Patients with Osteoporosis

**DOI:** 10.1155/2022/1447388

**Published:** 2022-09-15

**Authors:** Zhilan Fang, Shiyan Ouyang

**Affiliations:** ^1^First People's Hospital of Chenzhou City (Geriatric Comprehensive Ward Zone 1), Chenzhou, 423000 Hunan, China; ^2^First People's Hospital of Chenzhou City (General Surgery), Chenzhou, 423000 Hunan, China

## Abstract

Health monitoring can provide scientific and reasonable care for elderly users, professionally monitor the health parameters of the human body, and timely understand the user's own physical condition. By installing sensors with different functions in the rooms where the elderly often move and by installing vital signs sensors on their bodies, the data detected by the sensors are collected and analyzed in real time. Nursing refers to the fact that nursing staff must strictly follow the nursing system and operating procedures in the nursing work, accurately implement the doctor's orders, implement the nursing plan, and ensure that the patient is physically and mentally safe during treatment and recovery. Osteoporosis is a systemic bone disease in which bone density and bone quality are decreased due to various reasons, and the microstructure of bone is destroyed, resulting in increased bone fragility, which is prone to fractures. Osteoporosis is divided into two main categories: primary and secondary. Primary osteoporosis is divided into postmenopausal osteoporosis (Type I), senile osteoporosis (Type II), and idiopathic osteoporosis (including adolescent forms). This paper aims to study the healthcare effect of health monitoring system on elderly patients with osteoporosis, expecting to use the health monitoring system to provide more scientific care for the elderly and reduce the pain caused by osteoporosis. This paper proposes a study from the users of the elderly health monitoring products and the elderly home health products and analyzes the influencing factors of the usability design of the elderly home health monitoring system. This paper designs the overall framework of the elderly health monitoring system and designs the main components and application functions of the system. The experimental results in this paper show that there are 20 patients with osteoporosis due to lack of light, accounting for 16%. There are 10 patients with osteoporosis due to excessive coffee intake, accounting for 8%. There are 90 people who normally eat eggs, accounting for 75%, and 66 people who eat meat normally, accounting for 55%. According to the data, the health monitoring system can effectively control the diet of patients with osteoporosis.

## 1. Introduction

With the upgrading of science and technology, the living environment of human beings has been continuously improved, the level of medical facilities has also been continuously improved, and the society has experienced a low mortality rate. In addition to the improvement in medical care, the improvement in living conditions and economic and cultural development are the main reasons for the decrease in the mortality rate of the population. With the continuous change of fertility concept, low birth rate has also become a normal situation in society, which has also led to the accelerated arrival of population aging. As the aging situation continues to intensify, the healthcare of the elderly has also become a key social issue. It is very common for children to work in different places in society, which also increases the daily guardianship requirements of the elderly. The demand for healthcare in the lives of the elderly is also increasing, but there is a serious shortage of medical resources in China's nursing homes. Therefore, the construction of medical services for the elderly must keep up with the needs of modern elderly people, which is an inevitable requirement for social development. With the rapid development of smart devices, people's awareness of the Internet is getting higher and higher, and network monitoring is slowly appearing in life. In order to meet the needs of the market, a large number of health monitoring products have appeared on the market. However, these products have many deficiencies, and there is a large deviation from the physiological and behavioral needs of the elderly. In addition, traditional home health monitoring products only have a single function and do not have a systematic testing system; the usual monitoring does not have practical significance for the treatment of diseases or long-term observation results but only has the transient nature of monitoring the body indicators at the moment. So it is very necessary to study new health monitoring systems. Osteoporosis has a high probability in the elderly population, so it is very necessary to rely on the health monitoring system for osteoporosis care of the elderly.

RETRACTED

This paper takes the health monitoring system for the elderly as the research point and examines many issues to be considered in the design of home medical products for the elderly from the perspective of osteoporosis. It can promote the upgrading of monitoring products and improve the performance of products. Elderly people face many risk factors due to physical reasons, so it is very necessary to take care of the elderly, but it is normal for children not to be around due to work reasons. Therefore, using the health monitoring system to monitor the health of the elderly can reduce the burden on children and ensure the health of the elderly. The use of health monitoring systems can be effective in preventing chronic diseases in the elderly as their physical functions begin to decline and chronic diseases caused by diet and environment are more frequent.

This paper analyzes the daily activities of the elderly, which can monitor and display the physiological parameters of the elderly in real time and provide vital feature data for subsequent rescue; it relies on the powerful functions of the Android platform to send the measurement data to the remote health monitoring system through the GPRS network, which is convenient for the effective control of the data.

## 2. Related Work

As the proportion of the elderly increases, the society needs more and more medical resources for the elderly. In order to solve the shortage of medical resources, a health monitoring system for the elderly has emerged. Various current wireless health monitoring systems use the Internet of Things to transmit patient data through wireless sensor networks and then store and process the data through cloud computing. But using different types of wireless sensors on each system can lead to power efficiency issues. Nugraha B analyzed and compared the power consumption of six wireless health monitoring systems invented to monitor patient conditions and transmit data using wireless sensor networks. He analyzed three different technologies, namely, GPRS/UMTS (for one WHMS), Wi-Fi (for one WHMS), and Bluetooth (for four WHMSs). According to experiments, systems using Bluetooth as the transmission medium are more effective in reducing power consumption than other systems using GPRS/UMTS or Wi-Fi [1]. Through wireless sensor networks, it is possible to monitor the target area and identify the activities of the elderly through a large number of deployed sensor nodes. In addition, the limited energy supply of sensor nodes has become the biggest stumbling block, especially given the increasing size of the network, which is getting worse. Fu X provides an innovative energy-saving system based on energy-free RFID tags for monitoring the daily activities of the elderly to determine the physical condition of the elderly. The system realizes activity recognition by tracking passive RFID tags attached to the elderly based on the received backscattered signals [2]. Adequate healthcare is a major issue in many countries, especially underdeveloped and developing countries. The Internet of Things has a wide range of applications and has been applied in various fields such as security, intelligent transportation systems, smart cities, smart factories, and health. Kharel J focuses on the application of IoT in healthcare systems and proposes a new architecture leveraging IoT concepts under fog computing. The proposed architecture can be used to address the problems of clinic-centric health systems and transform them into patient-centric smart health systems [3]. Osteoporosis is a growing health problem worldwide, with complications as common as other common chronic diseases such as hypertension and diabetes. Alswat KA discusses the role of gender in osteoporosis, particularly in relation to peak bone mass and maturity, annual bone loss rates, screening, prevalence of osteoporosis and its associated fractures, osteoporosis post-fracture mortality, fracture risk prediction using different techniques, and the impact of gender on osteoporosis management [4]. Advances in information technology have witnessed tremendous advancements in healthcare technology in various fields today. However, these new technologies have also made healthcare data not only larger but more difficult. In order to provide a more convenient healthcare service and environment, Zhang Y proposes a cyber-physical system for patient-centric healthcare applications and services based on cloud and big data analysis technology, called Health-CPS. The results of this study suggest that cloud and big data technologies can be used to improve the performance of healthcare systems [5]. With the rapid development of the Internet of Things, cloud computing, and big data, more comprehensive and powerful applications emerge as the times require. Both advanced terminal technology and advanced cloud technology are expected to provide people with more reliable and intelligent services. Min C proposes a wearable 2.0 healthcare system to improve the QoE and QoS of next-generation healthcare systems. In the proposed system, a washable smart garment consisting of sensors, electrodes, and wires is a key component to collect user physiological data and receive the results of user health and emotional state analysis provided by cloud-based machine intelligence [6]. Population aging trends are a key global condition expected to have dire socioeconomic consequences for the population in the near future. Its contribution to the global burden of disease is increasing, and the implications of this situation for the future are awesome. Drawing on the researchers' experience and relevant literature, Asiamah N recommends a framework that will guide the development and institutionalization of a professional system of aged care, referred to here as affective aged care. The application of this framework by governments and healthcare organizations is expected to continue to improve care for the elderly as a means of healthcare management in response to aging [7]. Although these theories have discussed health monitoring systems and osteoporosis in the elderly to a certain extent, the combination of the two is less practical.

RETRACTED

## 3. The Role of Health Monitoring System in Healthcare of Elderly Patients with Osteoporosis

### 3.1. Health Monitoring System

In order to reduce the sudden symptoms caused by chronic diseases and prolong the life of the elderly, the treatment mode of chronic diseases for elderly patients has gradually shifted from long-term hospitalization to miniaturized family preventive treatment; this trend has led to the emergence of health monitoring products [8, 9]. Home health monitoring products have moved towards integration, using a combination of hardware and software, relying on hardware for a range of sign data collection and software for data analysis. Health monitoring is the use of scientific methods for physical and physical testing of the elderly. It studies the factors that produce changes and evaluates their reasons, gives suggestions for problems, and correctly gives specific implementation methods [10, 11].  Figure 1 shows the health monitoring systems that appear on the market:

Compared to the US monitoring system, China's monitoring system is immature, with more problems, professionalism of related products to be improved, lack of systematic operation, and an unsound market.

With the continuous upgrading of science and technology, people's requirements for health monitoring systems are becoming more and more diverse. Derived from a common sensor monitoring system to a wearable health monitoring system, the system is developed from wearable computers [12, 13]. Although wearable health monitoring products are new products, the concept of wearable monitoring has appeared in the 20th century. Compared with ordinary computers, the wearable monitoring system is more interactive and can provide users with private space [14, 15]. One of the smart wearable devices detects the movement of the body's joints and enables remote monitoring and supervision of patients who have undergone joint surgery, thus eliminating the need to go to hospital and allowing patients to complete their rehabilitation at home, saving hospital medical resources and patient treatment costs [16, 17]. The structure of the wearable monitoring system is shown in Figure 2:

Health monitoring systems can provide convenience for users in their lives, not only reducing medical expenses but also reducing the burden on children [18]. At present, large logarithmic children cannot take care of their parents all the time because of work needs. The health monitoring system can solve this problem, and this advantage also creates a market for the health monitoring system [19, 20]. Health monitoring systems provide patients with long-term professional care and enhance users' cognitive level and cognitive ability in self-monitoring and maintenance [21]. The device stores the collected data and location information in the computer, and analyzes and processes the data through special software, and finally forms a data analysis diagram for reference [22, 23].  Figure 3 shows the personalized health monitoring system.

RETRACTED

### 3.2. Wireless Location Technology

The most basic step of wireless sensor positioning technology is ranging. When the distance is measured, the unknown point can be estimated by relying on other equipment [24]. In the process of wireless positioning and ranging, we usually use the coordinate axis for calculation, as shown in Figure 4.

According to Figure 4, we can measure the distance of three points, as follows:

(1) $$\begin{array}{c} s_{1}=\sqrt{{\left(a-a_{1}\right)}^{2}+{\left(b-b_{1}\right)}^{2}}, \end{array}$$

(2) $$\begin{array}{c} s_{2}=\sqrt{{\left(a-a_{2}\right)}^{2}+{\left(b-b_{2}\right)}^{2}}, \end{array}$$

(3) $$\begin{array}{c} s_{3}=\sqrt{{\left(a-a_{3}\right)}^{2}+{\left(b-b_{3}\right)}^{2}}. \end{array}$$

Since the formula contains square values, there will be multiple solutions. But in practice, we only consider one set of solutions to calculate the position of the coincidence point [25].

(4) $$\begin{array}{c} \left(\begin{array}{c} a\\ b \end{array}\right)={\left(\begin{array}{c} 1.5\left(a-a_{1}\right)2.5\left(b-b_{3}\right)\\ 2.5\left(a_{2}-a_{3}\right)2.5\left(b_{2}-b_{3}\right) \end{array}\right)}^{-1.5}. \end{array}$$

Formula (4) represents the coordinates of the coincident points.

(5) $$\begin{array}{c} u\left(i\right)=\sqrt{u_{o}^{3}\left(i\right)+u_{l}^{3}\left(i\right)+u_{k}^{3}\left(i\right)}, \end{array}$$

where *u*(*i*) represents the output signal of the acceleration, and *u* represents the acceleration.

(6) $$\begin{array}{c} A_{i}=\int \frac{{\left|\bar{\alpha }\left(\delta \right)\right|}^{3}}{\delta }d\delta <\infty . \end{array}$$

Among them, $\bar{\alpha }\left(\delta \right)$ represents the Fourier transform, and *A*_*i*_ represents the value range of the Fourier transform. The Fourier transform represents the ability to represent a function satisfying certain conditions as a linear combination of trigonometric functions or their integrals [26, 27].

(7) $$\begin{array}{c} \alpha_{i,p}\left(p\right)=\frac{1}{\sqrt{g}}\alpha \left(\frac{p-\lambda }{g}\right), \end{array}$$

where *g* > 0, *a* represent the scale factor, and *λ* represents the translation factor.

RETRACTED

As shown in Figure 5, the point in the upper right corner is the unknown point, and the *Q* point is the known point, and the distance between the two points is *b*; we can get:

(8) $$\begin{array}{c} b=\sqrt{{\left(a-a_{1}\right)}^{2}+{\left(b-b_{1}\right)}^{2}+{\left(c-c_{1}\right)}^{2}}, \end{array}$$

(9) $$\begin{array}{c} \eta =\arctan\frac{b-b_{1}}{a-a_{1}}, \end{array}$$

(10) $$\begin{array}{c} \phi =\arccos\frac{c-c_{1}}{b}. \end{array}$$

If there is interference in the external environment when measuring the distance, we need to change the calculation method:

(11) $$\begin{array}{c} g_{1}\left(a,b,c\right)=\sqrt{{\left(a-a_{1}\right)}^{2}+{\left(b-b_{1}\right)}^{2}+{\left(c-c_{1}\right)}^{2}}, \end{array}$$

(12) $$\begin{array}{c} g_{2}\left(a,b,c\right)=\arctan\frac{b-b_{1}}{a-a_{1}}, \end{array}$$

(13) $$\begin{array}{c} g_{3}\left(a,b,c\right)=\arccos\frac{c-c_{1}}{b}. \end{array}$$

Assuming that the errors are independent random variables, the conditional probability function expression is as follows:

(14) $$\begin{array}{c} w=\frac{1}{\sqrt{{\left(3\pi \right)}^{2.7}\prod_{1}^{2.7}\beta_{j}}}\exp\left(-\overset{2.7}{\underset{1}{\sum }}\frac{1}{2\beta_{j}^{2}}{\left(d-j\right)}^{2}\right). \end{array}$$

According to the above formula, the coordinates in the figure can be obtained as:

(15) $$\begin{array}{c} b_{1}=\frac{1}{\det\left(w\right)}\left(w_{4}w_{5}-{w_{3}}^{2}\right), \end{array}$$

(16) $$\begin{array}{c} b_{2}=\frac{1}{\det\left(w\right)}\left(w_{1}w_{5}-{w_{2}}^{2}\right), \end{array}$$

(17) $$\begin{array}{c} b_{3}=\frac{1}{\det\left(w\right)}\left(w_{1}w_{4}-{w_{2}}^{2}\right). \end{array}$$

According to the calculation, when calculating the geometric distance between the target objects, it has a great relationship with the angle between the objects.

(18) $$\begin{array}{c} SNR=13\log\frac{\sum a^{3}\left(p\right)}{\sum_{p}^{W}\delta^{3}\left(p\right)}. \end{array}$$

*a*(*p*) represents the standard limit number, *δ*(*p*) represents the noise signal, and *W* represents the signal length.

(19) $$\begin{array}{c} \alpha_{r,i}\left(x\right)=u_{1}^{-r/3}\alpha \left(u_{1}^{-r}-h\varepsilon_{1}\right), \end{array}$$

where 1 stands for discrete wavelet.

(20) $$\begin{array}{c} \alpha_{r,i}\left(x\right)=3^{-r/3}\alpha \left(3^{-r/3}p-h\right), \end{array}$$

where 1, 2.

### 3.3. Overview of Osteoporosis

Osteoporosis is a disease of the skeletal system characterized by a decrease in bone density and an increased risk of fracture [28]. From the current research, with the increase of age, the probability of suffering from osteoporosis is greater [29]. Symptoms of osteoporosis include painful patients may have low back pain or peripheral aches, spinal deformities osteoporosis may be severe with shortening of height and hunchback as well as fractures non-traumatic or minor trauma occurring as fragility fractures. With the prolongation of lifespan and the deepening of population aging, the phenomenon of osteoporosis in society is becoming more and more common, and osteoporosis has become an important health problem for human beings [30, 31].

RETRACTED

There are many reasons for osteoporosis. According to the survey, long-term unreasonable dietary factors are the most common and controllable factors [32]. Uncontrollable factors in osteoporosis include race and genetics, age and sex, and the number of births. Failure to establish optimal peak bone mass in young adults and excessive bone loss rate in later stages can lead to the occurrence of osteoporosis, both of which can be improved by a reasonable diet. Increasing the control of controllable factors in the elderly can alleviate the symptoms of osteoporosis [33, 34]. The pain itself can reduce the patient's quality of life. Spinal deformities and fractures can be disabling, leaving the patient with limited mobility, unable to care for themselves, and increasing the incidence of lung infections and bed sores.  Figure 6 is a schematic diagram of the causes of osteoporosis:

## 4. Experiment on the Healthcare Effect of Health Monitoring System on Elderly Patients with Osteoporosis

### 4.1. Experimental Subjects

In this experiment, the elderly osteoporosis situation was investigated in the B district of A city. A total of 120 subjects were included in this experiment, and the details are as follows.

According to the data in Table 1, in this questionnaire, there are 55 men with osteoporosis, accounting for 45.8% and 65 women with osteoporosis, accounting for 54.2%. In terms of age, 22 osteoporosis patients were younger than 50 years old, accounting for 18.3% and 98 patients were older than 50 years old, accounting for 81.7%. According to the data, from the perspective of gender of osteoporosis patients, female patients are more likely to suffer from osteoporosis; judging from the age of the patients, the group over 50 has a higher probability of developing osteoporosis, but the group under the age of 50 still has the possibility of developing osteoporosis.

According to the data in Table 2, among the subjects of this experiment, 43 people have a college degree or above, accounting for 35.8%; 65 people have a middle school diploma, accounting for 54.2%; 12 people have a primary school diploma, accounting for 10%. In terms of marital status, 59 of the patients with osteoporosis were married, accounting for 49.1% and 61 of the patients were divorced or widowed, accounting for 50.9%. According to the data, there was no significant relationship between osteoporosis patients and marital status and diploma.

RETRACTED

### 4.2. Knowledge of Osteoporosis among Survey Respondents

Osteoporosis is very common in daily life. In order to understand the situation of osteoporosis patients in daily life, we conducted the following knowledge survey on osteoporosis patients. The details are as follows.

According to the data in Table 3, according to the scores of the experimental subjects, in terms of calcium knowledge, the highest score is 7 points, the lowest score is 0 points, and the average score is 3.5; in terms of sports knowledge, the highest score is 9 points, the lowest score is 1 point, and the average score is 5; in terms of dangerous situations, the highest score is 8 points, and the lowest score is 1 point, and the average score is 4.5. According to the data, the average score of calcium knowledge is the lowest, and the average score of exercise knowledge is the highest. Relatively speaking, osteoporosis patients have a better understanding of exercise knowledge and lack of calcium knowledge, but calcium knowledge is more important for osteoporosis. Therefore, it is necessary to increase the public's understanding of calcium knowledge.

### 4.3. Occupational Situation of Patients with Osteoporosis

In order to study the etiology of osteoporosis patients, we investigated the occupations of osteoporosis patients, as follows.

According to the data in Table 4, among the osteoporosis groups surveyed, 9 people are farmers, accounting for 7.5%; 57 people are workers, accounting for 47.5%; 12 people are cadres, accounting for 10%; 15 people are cadres, accounting for 10%; people are self-employed, accounting for 12.5%; 25 people are other occupations, accounting for 22.5%. According to the data, among the surveyed groups, the occupation with the highest probability of suffering from osteoporosis is the worker, followed by the self-employed. Due to the long-term single labor in the factory, workers are more tiring and have less time to exercise, which is prone to osteoporosis.

## 5. The Healthcare Effect of Health Monitoring System on Elderly Patients with Osteoporosis

### 5.1. Health Questionnaire before and after Health Monitoring System Testing

Good health is the pursuit of osteoporosis patients. In order to confirm the effect of the health monitoring system, we conducted a health survey analysis of the patients, including physiological function (PF), physiological function (RP), general health status (BP), social function (SF), health vitality (GH), vitality (VT), mental health (MH), and emotional role (RE) eight dimensions. The details are as follows:

According to the data in Figure 7, before the experiment, we divided the osteoporosis patients into two groups. The control group did not use the health monitoring system, and the experimental group used the health monitoring system. Before the experiment, we conducted a health survey on the two groups of patients. Among them, the average physical function of the control group was 80 points, the physiological function was 76 points, the overall health was 82 points, the social function was 59 points, the health vitality was 57 points, the overall vitality was 55 points, the mental health was 63 points, and the emotion was 63 points. The role is 78 points; the emotional role is 78 points. The patients in the experimental group had an average of 78 points for physiological function, 76 points for physiological function, 81 points for overall health, 60 points for social function, 58 points for health vitality, 53 points for overall vitality, 62 points for mental health, and 80 points for emotional role. According to the experimental data of the two groups, the overall conditions of the two groups of patients before the experiment were not much different, and there was no other impact on the subsequent experiments.

RETRACTED

The next step is to analyze the nursing situation of the two groups of patients. Osteoporosis patients without health monitoring system care scored an average of 67 points for physiological function, 60 points for physiological function, 76 points for overall health, 57 points for social function, 50 points for health and vitality, and 55 points for overall vitality, mental hygiene scored 57 points and emotional roles scored 79 points. The average physiological function of osteoporosis patients nursing through the health monitoring system is 80 points, the physiological function is 78 points, the overall health is 74 points, the social function is 60 points, the health vitality is 61 points, the overall vitality is 65 points, and the mental health is scored 61 points. the emotional role is 81 points, the mental hygiene is 65 points. According to the data, patients who did not receive healthcare showed a significant decline in social functioning and health vitality. There were varying degrees of decline in other areas, while osteoporosis patients with professional care remained generally well. These data suggest that patients with osteoporosis require specialized care to maintain normal levels.

According to the data in Figure 8, in order to explore the control of high-risk conditions of osteoporosis patients by the health monitoring system, we conducted a comparative analysis of the two groups of patients. There was no significant difference in the high-risk exercise frequency between the two groups of osteoporosis patients before the experiment. The osteoporosis patients in the control group did not receive health monitoring system care, and the experimental group received healthcare. In the control group, 84 patients lacked exercise, accounting for 70%; 73 patients suffered from osteoporosis caused by consuming soy products, accounting for 61%; 48 patients suffered from osteoporosis caused by consuming dairy products, accounting for 40%. There are 64 patients with osteoporosis due to sedentary, accounting for 53%; 32 patients with osteoporosis due to smoking, accounting for 27%; 24 patients with osteoporosis due to drinking, accounting for 20%; there are 42 patients with osteoporosis due to lack of light, accounting for 35%; 30 patients with osteoporosis due to excessive coffee intake, accounting for 25%. There were 40 patients in the experimental group who lacked exercise, accounting for 33%; there are 36 patients with osteoporosis caused by the intake of soy products, accounting for 30%; 20 patients with osteoporosis caused by the intake of dairy products, accounting for 17%; there are 32 patients with osteoporosis due to sedentary, accounting for 27%; 36 patients with osteoporosis due to smoking, accounting for 30%; 18 patients with osteoporosis due to drinking, accounting for 15%; there are 20 patients with osteoporosis due to lack of light, accounting for 16%; 10 patients with osteoporosis due to excessive coffee intake, accounting for 8%. Based on this data, patients who were cared for by the health monitoring system showed a significant improvement in the frequency of high-risk conditions. The frequency of high-risk conditions is higher in patients who do not receive professional care, so health monitoring systems can help reduce osteoporosis symptoms.

RETRACTED

### 5.2. Dietary Structure of Patients

A balanced dietary structure is very important for human health, so maintaining a scientific and reasonable dietary structure for patients with osteoporosis is conducive to maintaining good health.

According to the data in Figure 9, in order to explore the control of the health monitoring system on the diet of patients with osteoporosis, we conducted a comparative analysis of the two groups of patients. And there was no significant difference in the diet of the two groups of osteoporosis patients before the experiment. The osteoporosis patients in the control group did not receive health monitoring system care, while the experimental group received healthcare. In the control group, 76 people had a normal intake of vegetables, accounting for 63%; 60 people had a normal intake of fruits, accounting for 50%; 58 people normally ingest fish and shrimp, accounting for 49%; 66 people normally ingest eggs, accounting for 55%; 54 people normally ingest meat, accounting for 45%; there were 80 people who normally ingest dairy products, accounting for 67%, 53 people who normally ingested oils and fats, accounting for 44%, and 47 people who ingested salt normally, accounting for 39%. In the control group, 102 people had a normal intake of vegetables, accounting for 85%; 92 people had a normal intake of fruits, accounting for 77%; 84 people normally ingest fish and shrimp, accounting for 70%; 90 people normally ingest eggs, accounting for 75%; 66 people normally ingest meat, accounting for 55%; there were 98 people who normally ingest dairy products, accounting for 82%; 84 people who normally ingested fats and oils, accounting for 70%; 78 people who ingested salt normally, accounting for 65%. According to the data, the health monitoring system is beneficial to know the dietary intake of patients with osteoporosis and can better achieve the nursing effect.

### 5.3. Nutritional Intake of Patients

The physical function of the elderly begins to decline, and the energy needed by the body needs to be replenished in time. However, the nutrients the body needs are not as good as possible, and scientific and reasonable intake is required.

According to the data in Figure 10, in order to explore the nutritional intake of patients with osteoporosis by the health monitoring system, we conducted a comparative analysis of the two groups of patients. Before the experiment, the protein intake of osteoporosis patients in the control group was 15.33 g, and the protein intake after general nursing was 14.7 g; vitamin A intake was 297 *μ*gRE and post-general care intake was 305 *μ*gRE; vitamin C intake was 57 mg, and 54 mg after general nursing; calcium intake was 515 mg, and 507 mg after general nursing; phosphorus intake was 202 mg and post-general care intake was 187 mg; zinc intake was 4.5 mg and post-general care intake was 4.03 mg; magnesium intake was 205 mg, 205.7 mg after general nursing; dietary fiber intake was 18 g, and 17.06 g after general nursing. Based on this data, general care did not significantly change the nutritional intake of patients with osteoporosis.

Before the experiment, the protein intake of osteoporosis patients in the experimental group was 16 g, and the protein intake after general nursing was 4 g; vitamin A intake was 297 *μ*gRE and post-general care intake was 230 *μ*gRE; vitamin C intake was 54 mg and post-general care intake was 43 mg; calcium intake was 507 mg and post-general care intake was 320 mg; phosphorus intake was 202 mg and post-general care intake was 187 mg; zinc intake was 4 mg and 3 mg after general care; magnesium intake is 200 mg, and after general care intake is 105 mg; the dietary fiber intake was 18 g, and the intake after general care was 12 g. According to the data, health monitoring system nursing has a significant trend of reducing the nutritional intake of patients with osteoporosis.

RETRACTED

There was no significant difference in diet between the two groups of osteoporosis patients before the experiment. The osteoporosis patients in the control group did not receive health monitoring system care, and the experimental group received healthcare. Osteoporotic patients who received professional care showed significant improvements in nutritional intake closer to normal levels.

## 6. Conclusions

With the advancement of science and technology and the improvement of economic level, people's living standards are also constantly improving, and more attention has been paid to physical health. At present, the aging situation in China is relatively serious, the proportion of the elderly is increasing, and the elderly need more medical resources. This paper aims to study the healthcare effect of health monitoring system on elderly patients with osteoporosis, expecting to use the health monitoring system to provide more scientific care for the elderly and reduce the pain caused by osteoporosis. The main findings of this paper are as follows: (1) Patients with osteoporosis who have undergone specialist care have shown significant improvements in nutritional intake, which is closer to normal levels. (2) The health monitoring system facilitates the knowledge of the dietary intake of osteoporotic patients and allows for better care outcomes. Although this paper has achieved certain results, there are still many shortcomings: (1) Among the detection nodes of this system, the nodes involved in health index detection are mainly body temperature detection nodes. Relatively speaking, it can also add multiple detection modules such as blood pressure, heart rate, and blood sugar to enrich the functions of the system. (2) The scope of research on elderly users is still relatively narrow. Most of the research data feedback information of elderly users comes from the urban elderly, which cannot represent all the elderly.

## Figures and Tables

**Figure 1:** Routine health monitoring system.

**Figure 2:** Structure of wearable monitoring system.

**Figure 3:** Personalized health monitoring system.

**Figure 4:** Coordinate axis measurement.

RETRACTED

**Figure 5:** Angle and distance.

**Figure 6:** Architecture of symptoms that trigger osteoporosis.

**Figure 7:** Analysis of health questionnaires before and after monitoring.

**Figure 8:** Comparison of high-risk situations.

**Figure 9:** Dietary structure analysis.

**Figure 10:** Analysis of patient nutritional intake.

**Table 1:** Basic information of experimental subjects.

Projects		Number of people	Proportion (%)
Gender	Male	55	45.8
	Female	65	54.2

Age	Less than 50 years old	22	18.3
	Over 50 years old	98	81.7

**Table 2:** Information about the experimental subjects.

Projects		Number of people	Proportion (%)
Education level	Post-secondary	43	35.8
	Secondary	65	54.2
	Primary school	12	10

Marital status	Married	59	49.1
	Divorced or widowed	61	50.9

**Table 3:** Osteoporosis knowledge scores.

Category	Highest score	Lowest score	Average score
Calcium knowledge	7	0	3.5
Exercise knowledge	9	1	5
Dangerous conditions	8	1	4.5
Total score	24	2	13

**Table 4:** Occupation of patients with osteoporosis.

Category	Number of people	Proportion (%)
Farmers	9	7.5
Workers	57	47.5
Cadres	12	10
Individuals	15	12.5
Others	25	22.5

## Data Availability

This article does not cover data research. No data were used to support this study.
